# A Study on the Impact of Wushu Sports Health on College Students' Mental Health

**DOI:** 10.1155/2022/5841017

**Published:** 2022-08-29

**Authors:** Yijia Sun, Bo Zhang, Aijun Ji, Wei Sun

**Affiliations:** ^1^Jining Medical University, Jining, Shandong, China; ^2^Weifang Middle School, Weifang, Shandong, China

## Abstract

At the current university stage, university students are subjected to a variety of pressures such as role change adaptation pressure, study and life pressure, emotional pressure, economic pressure, employment pressure, and interpersonal pressure, which seriously affect their physical and mental health. Students with poor psychological tolerance may develop psychological disorders and, in serious cases, may even lead to mental illness. The results of the study indicated that 17%–20.23% of university students have psychological disorder problems. Excessive and long-lasting stress can cause psychological, depression and anxiety, physical fatigue, and discomfort, which can lead to various diseases and even death. It is, therefore, of great importance to study the state of mental health and stress among university students as well as to develop countermeasures to improve their mental health. This study focuses on the impact of martial arts sports on the mental health of university students. As a type of sport, martial arts sports are particularly special in which they can intertwine the nurturing spirit of traditional culture with the nurturing spirit of sports. The development of martial arts sports in colleges and universities can not only enhance the physical quality of college students but also promote the development of their physical and mental health. Therefore, this article takes Taijiquan as an example to explore the study of the impact of martial arts sports health on college students' mental health.

## 1. Introduction

As far as the formation of a healthy personality in students is concerned, physical education stands out and is special in its unique form, rich content, and positive pedagogical function, which cannot be matched by other disciplines. The main objective of university physical education is to promote the health of students. Health is not only superficially physical, but also includes mental health, social adaptability, and moral health (i.e., personal health), and only the harmonious and coordinated development of body and personality is true health in this sense [1]. Physical education consists mainly of physical training, which is very practical. Physical training is not only physically useful but is accompanied by factors such as knowledge and information, mental activity, and emotional experience. Therefore, physical education at the right time and in the right context is twice as effective and can be very beneficial in shaping a healthy personality in students [2]. The current health status of students is not good; usually, they do not have nutritional deficiencies or serious health problems, but what they lack most is a healthy lifestyle. If they are aware that their habits, emotions, social environment, personality, and character can affect their health and well-being in their daily lives, and if the school can provide them with facilities for outdoor activities, they will choose the “sport” approach to improve their health. In school sports, the martial arts programme is representative of traditional Chinese sports. Eastern sports, represented by traditional Chinese sports, and modern Western sports belong to two major sports systems that are vastly different. The origins of Eastern sports are closely linked to traditional mythology, religious rituals, and warfare, and the obvious factors that play a major dominant role are ancient Eastern philosophy and ethics. The direct aim of the exercise is “for one's own sake,” to achieve one's own goals, to benefit oneself, for one's own “health,” and “longevity,” while the indirect aim is social. In terms of the means of exercise, the emphasis is not on “practice” [3], but on “nourishment,” combining nourishment and practice. The practice emphasizes “moderation and proportionality” is appropriate to the person and the time; is not excessive; meets the needs of the human body for “health” and “longevity”; is not too concerned about competition and victory; is steady, self-indulgent, safe, and pays attention to social norms; advocates “observing its virtue” with rituals and “observing its rituals” with the body. In terms of social and educational purposes, the East incorporates moral education into sports and applies ethical concepts such as “benevolence” [4] “love,” “ritual,” and “let” to the norms of sports, emphasizing a holistic view of human health, advocating “making the body evenly developed,” and “suppressing its faults while saving its shortcomings.” From a theoretical point of view, it attaches importance to the medical and philosophical research required for health and longevity and applies the theory of “the unity of heaven and man” as a guiding principle [5].

In the new century, with the development of society, the rapid growth of the economy, the expansion of information, the intensification of competition, and the pressure of employment, university students not only need higher knowledge and skills but also need a healthy body to adapt to the needs and guarantees of society. A healthy body for university students is vital for employment and better work, and martial arts not only improves the physical fitness of university students but also improves mental health and has the function of promoting socialization [6]. Wushu programmes are representative of all general university sports, whether they are large or small traditional sports. Wushu has the unique advantage that it helps to shape and develop the character of students. Wushu programs have a rich and unique form of practice that is closely related to the content and cultural characteristics of students' healthy personality traits.

Taijiquan is a traditional Chinese martial art that has long been used as a training and fitness tool at home and abroad. In this study, we have taken Taijiquan as an example to explore the impact of traditional martial arts on the mental health status of university students. Nowadays, there are many different types of movements and routines in Taijiquan, such as Chen, Yang, Wu, and Sun. Nevertheless, the different types of exercises and training routines have common features and similar training effects on the human body [7]. Among them, the Simplified Taijiquan 24 Form is popular among Taijiquan practitioners because it has standardized and unified movements. It is a set of Taijiquan exercises selected by the State General Administration of Sports in 1956 to popularize Yangqi Taijiquan. It follows the main features of traditional Taijiquan and is very popular among Taijiquan practitioners, especially beginners, abroad [8].

Due to the differences between the East and West in terms of philosophical underpinnings of fitness, sociocultural, ethnic, and religious beliefs, different forms of fitness can have different effects on the physical and mental health of young people, and studies have shown that rhythmic repetitive exercise such as swimming can have a psychological impact. However, young people should explore the benefits of traditional forms of physical activity on their physical and mental health as well as the physical and mental effects of different programmes. The use of martial arts teaching in compulsory education to improve the physical and mental health of students while fostering a good national spirit is a special need for character education in schools; the use of optional martial arts courses to educate students about healthy personalities is an important topic for physical education in colleges and universities, and an in-depth study of this topic from a theoretical perspective could help to enrich and improve the theory on the one hand. From a practical point of view, it will help to recognize the importance of using traditional sports to cultivate a healthy personality, clarify the role of Wushu programmes, which are an important part of traditional national sports, in cultivating a healthy personality among university students [9], recommend students with different needs to Wushu programmes that meet their characteristics, help to strengthen the elements of a healthy personality, and fully exploit the special role of Wushu programmes in universities. This article examines the impact of a martial arts programme on the healthy personality of university students through their voluntary participation in a martial arts programme [10, 11].

## 2. Objectives and Research Methodology

The subjects of this study were university students. Thirty students were selected from each of the two classes of the School of Physical Education of a university in the class of 2021, making a total of 60 students. The average age of the subjects was 22 ± 1.5 years. The experimental subjects were all able-bodied, had no major illnesses, and had not practiced Taijiquan before. The subjects will be divided into an experimental group and a control group. The subjects in the experimental group would be trained in Taijiquan for a period of 4 months (16 weeks in total), while the subjects in the control group would be strictly controlled not to practice fitness Qigong and would be used to compare with the subjects in the experimental group in order to study the effect of Taijiquan on the mental health of university students [12–15].

An experimental intervention was developed and applied to the study sample for 4 months. A pretest was provided to both groups prior to the start of the experiment, and a posttest was administered 4 months later to obtain pretest and posttest data for both groups.

The SCL-90 scale (version 1–5 items) was used in the experiment. Scores for each factor were compared between the two study groups to determine significant differences.

The data and information obtained was computer generated using Excel and entered into a database. SPSS 18.0 software was used to process and analyse the data, and *t*-tests were used to compare the means to see if there were significant differences between the data. The questionnaires were categorized and valid questionnaires were numbered after excluding invalid questionnaires [16, 17]. A database was created using Epidata 3.0 software, and statistical processing was carried out using SPSS 19.0 software. Descriptive statistics, *t*-test, *Z*-test, ANOVA, correlation analysis, regression analysis, and chi-squared test were used to analyse the study data. The correlation methods were defined and communicated as follows: *Z*-test: Let *x*1, *x*2,…,*n* be a sample of capacity *n* taken from the normal overall N(*μ*), *x* and S are the sample mean and sample variance, respectively, with known constants greater than 0. The following are the *U* tests for the unknown parameter *μ*, respectively: *s*^2^ = *σ* is known, test H_0_: *µ* = *μ*_0_, H_1_: *μ* ≠ *μ*_0_. Choice of statistic:

(1) $$\begin{array}{c} u=\frac{\bar{x}-\mu_{0}}{\sigma_{0}}\sqrt{n}. \end{array}$$

Under the assumption that H holds, *u* obeys the N(0, 1) distribution, and for a given significance level a, checking the standard normal distribution table yields the critical value *u*_*a*_ such that:

(2) $$\begin{array}{c} P\left(\left|u\right|\geq u_{a/2}\right)=\alpha ,\\ A=\left\{\left|u\right|\geq u_{a/2}\right\}. \end{array}$$

The correlation coefficient formula is as follows:

(3) $$\begin{array}{c} r\left(X,Y\right)=\frac{\text{Cov}\left(X,Y\right)}{\sqrt{\text{Var}\left[X\right]\text{Var}\left[Y\right]}}. \end{array}$$

The Pearson coefficient in the chi-squared test is calculated as follows:

(4) $$\begin{array}{c} \chi^{2}=\sum_{i=1}^{k}\frac{{\left(f_{i}-np_{i}\right)}^{2}}{np_{i}}. \end{array}$$

### 2.1. Design and Operation of the Experiment

Sampling: The two groups of subjects, the experimental group and the control group, should be as similar as possible in all conditions except for the experimental control. The author used the students of two classes of the School of Physical Education of a university in the class of 2021 as the sampling subjects. Through comparison, it was found that the students of the two classes were similar in terms of age, physical condition, and curriculum situation and that all students were in good health, had sound limbs, had no major illnesses, and had no previous exposure to Taijiquan; it was also learned through visits to the grade office that the entrance classification of the 2021 social sports class was completely random, and there was no case where the overall entrance performance of one class was better than that of the other class, so it was determined that the students of the two classes were similar in terms of age, physical condition, and course scheduling situation. Paired random sampling was used to divide all subjects into two groups, male and female, and a sample of 30 cases was randomly selected from each group by lottery, that is 30 male cases and 30 female cases [18].

Grouping: The sample of 60 cases drawn was divided into two groups, namely the experimental group and the control group. In the grouping, 15 male students were randomly selected from the total sample by means of a two-colour. In the grouping, 15 boys and 15 girls were randomly selected as the experimental group and the remaining 15 boys and 15 girls as the control group.

Procedure of the experiment: The subjects in the experimental group were arranged to practice Taijiquan twice a week, on Tuesday and Thursday mornings, outside of class time, for 1.5 h each time, from 9:00am to 10:30am. The same fitness Qigong instructor coached and instructed the subjects in the experimental group for a period of 4 months (16 weeks in total). The experiment was conducted in an orderly manner under the supervision of the researcher. The subjects in the experimental group learned to practice Taijiquan under the guidance of the fitness Qigong instructor. The training of the experimental subjects was divided into two parts—the training of gongfu and the teaching of theory. The theoretical teaching was mainly to explain the principles of fitness Qigong, the types of fitness Qigong, the origin and development of Taijiquan, and the characteristics and movements of Taijiquan to the subjects in the experimental group. Theoretical teaching time does not take up training time. The teaching of gongfu is mainly to teach the experimental subjects the new Taijiquan routine, to solve their doubts, to correct the wrong movements, and to explain the main points of the gongfu movements to ensure that each subject can practice Taijiquan with the most standard posture. Before each practice session, a review of what has been learned is given, and the instructor corrects any errors or redundant movements at this time, ensuring that their movements are automated after several repetitions. Each time the exercises will be accompanied by special practice music. The instructor will lead each exercise in front of the group for the first time, and then the subjects will practice on their own while the instructor corrects them. The 1.5 h of each exercise will be divided into the following parts.

1. The first 20 min: roll call to ensure that the subjects are present and then organize the subjects in the experimental group to practice Taijiquan, with the instructor leading the practice
2. 20 min–35 min: the experimental subjects are rested and relaxed
3. 35 min–65 min: the experimental subjects continue to contact Taijiquan, with the instructor on hand to correct them
4. 65 min–80 min: the experimental subjects are rested, recuperated, and relaxed
5. 80 min–90 min: the subjects in the experimental group performed the last exercise, led by the instructor

After the researcher finished taking attendance of the experimental group to ensure that no subject left early, the group was dismissed.

Taijiquan is a bionic gongfu method that emphasizes the combination of movement and stillness, and the coexistence of rigidity and flexibility, which helps to harmonize the internal and external harmony of the practitioner's torso. The movements and the mood of Taijiquan are an inseparable whole, and ignoring one or the other will not bring out the full effect of Taijiquan. It can be said that the idea of forming the body as a whole is the integration of the concept of harmonizing the body, the form, and the spirit. It is not enough just to be like the form of Taijiquan movements, but also to be like the spirit, to feel oneself as one with the five birds, and to feel oneself as one with nature. This is the only way to put aside distracting thoughts and achieve the goal of Taijiquan fitness and mindfulness.

Before the start of the experiment, a pretest was organized for all subjects in the experimental and control groups in the step classroom. Members of the experimental and control groups were seated randomly, with an empty seat between every two subjects. The researcher handed out the SCL-90 scale and the pens to be used to fill it out and explained how to fill it out. Each question was graded on a scale of 5, with 1 being not at all and 5 being very severe. The scale took 1 hour to complete and was collected at the end of the hour. All subjects were not allowed to talk to each other or look at their mobile phones while completing the scales, and the whole process was supervised by the researcher. The pen was given to the participant as a souvenir and a snack was given to the participant as a gift after completing the scale. If subjects completed the scales within 1 hour, they were still not allowed to talk to others or look at their mobile phones, and the process was supervised by the researcher until all scales were collected after 1 hour.

The posttest process was basically the same as the pretest. At the end of the experiment, the posttest was administered to all subjects in the experimental and control groups in the classroom (same location as the pretest). Members of the experimental and control groups were seated randomly, with an empty seat between every two subjects. The researcher (coach, author) handed out the SCL-90 scale and the pen to be used to fill it out and again explained how to fill out the scale. The instructions were generally that there were 90 questions on the SCL-90 and each participant was asked to fill in the questions based on their own experiences over the last 2 weeks. Each question is graded on a 5-point scale, with 1 being not at all and 5 being very severe. The scale was to be completed in 1 hour and collected at the end of the hour. All subjects were not allowed to talk to each other or look at their mobile phones while completing the scale. To ensure the validity of the scale data, the whole process of completing the scale was counted as a regular grade and recorded as a final grade. Subjects who completed the scales within 1 hour were still not allowed to talk to others or look at their mobile phones. After the posttest, the researcher thanked the subjects and gave each subject a drink as a small gift.

Subjects in the experimental group were asked not to concentrate on practicing any other kind of fitness Qigong in any form during the experiment except the Taijiquan they practiced during the experiment; subjects in the control group were asked not to concentrate on practicing any form of fitness Qigong during the experiment. Since the subjects in both the experimental and control groups belonged to different classes in the same school, and their curricula and settings were almost the same, it could be introduced that the objective conditions affecting the subjects in the two groups were basically the same in their ordinary school life, so not too much control was done. In other words, the objective life and study conditions of the subjects in the two groups are basically the same, except for the experimental training of the subjects in the experimental group after school hours.

I hypothesize that Taijiquan can improve the mental health of university students and can significantly improve the factors of “depression” and “anxiety.” There is no significant difference in the total scores between men and women.

## 3. Results and Analysis of the Experiment

### 3.1. Homogeneity Test of the Experimental and Control Groups

As can be seen from Table 1, there was no significant difference between the subjects in the experimental and control groups, which came from the same whole. The Sig values for all ten factors were greater than 0.05 (*p* > 0.05), which would indicate that there was no significant difference between the two groups at the time of the pretest, that is the subjects in the experimental and control groups were all comparable in their level of mental health when they were grouped together, and there was no situation where one group was significantly better on one factor than the other. Looking at the factor scores for each factor, the average factor score for subjects in both groups was less than 2, demonstrating that subjects in both groups had a better average in these ten areas and had no significant mental illness. However, individual subjects in both groups scored more than 2 on the “obsessive-compulsive symptoms” factor, and individual subjects in the experimental group scored more than 2 on the “other” factor, indicating that these subjects had some psychological disorders in these factors, and their mental health in these areas needs to be improved.

### 3.2. Intergroup Comparison of Posttest in the Experimental Control Group

As can be seen from Table 2, there are significant differences between the subjects in the experimental and control groups. The factors that were significantly different were: depression, anxiety, and hostility, with particular significance in the two factors of depression and anxiety. There were no significant differences in the total scores of the two groups. The SIG value for the depression factor and anxiety factor was 0.001 (*p* ≤ 0.01) and 0.000 (*p* ≤ 0.01), respectively, indicating that on these two factors the experimental control group differed significantly. The mean score for depression was 14.57 in the experimental group and 16.23 in the control group, indicating that the experimental group was significantly better than the control group in terms of depression; the mean score for anxiety was 11.87 in the experimental group and 14.23 in the control group, indicating that the experimental group was also significantly better than the control group in terms of anxiety. In terms of depression, the per capita factor score of subjects in the experimental group was 1.12 ± 0.14 and that of subjects in the control group was 1.25 ± 0.14, neither of which was higher than 2, indicating that there was no psychological disorder in depression in the two groups. In terms of anxiety, subjects in the experimental group had a per capita factor score of 1.19 ± 0.14, and those in the control group had a per capita factor score of 1.42 ± 0.12 which was lower than 2. Moderate exercise, stress relief, and interaction with others are all effective means of treating depression and anxiety, and the practice of tai chi has these effects. Before practicing Taijiquan, one is required to eliminate distracting thoughts and concentrate on the Dantian, while when practicing Taijiquan, one is required to enter the state of mind, breath, and form, which can effectively relieve the stress of the subjects.

The SIG value for the hostility factor was 0.046 (*p* ≤ 0.05), indicating that there was a significant difference in the hostility factor between the experimental group and the control subjects. The mean score of the experimental and control subjects was 7.23 and 8.13, respectively, indicating that the experimental subjects were significantly better than the control subjects. The per capita factor score of the subjects in the experimental group was 1.21 ± 0.25 and that of the subjects in the control group was 1.36 ± 0.32, which was less than 2, indicating that the subjects in the experimental and control groups did not have mental illness in terms of hostility. By improving the subjects' mindset, enhancing their harmony and unity with nature, and improving the communication between the subjects and the coach, and between the subjects and the subjects, the practice of Taijiquan improved their level of hostility, making the overall level of the experimental group in this aspect significantly better than that of the control group.

### 3.3. Intragroup Comparison of Pretest and Posttest in the Control Group

Table 3 shows the comparison between the pretest and posttest data of the control group. It is easy to see that although there was a change in the levels of the pre- and posttests in the control group, the change did not reach significance. The *P*-values for all ten factors in the control group were greater than 0.05, demonstrating that there was no significant difference. In terms of mean values, the mean values of all the factors except for the “terror” factor decreased, but the changes were not significant and did not reach significance, so such changes were negligible. The reason for the small difference between the posttest and pretest scores of the control group is that the control group was strictly controlled not to participate in taijiquan learning and exercise, and all the subjects in the control group did not participate in activities that could interfere with their mental health, and during the experimental period, they went about their daily lives and studies as usual, so there was not much change in their state of mind between the pretest and the posttest, and their total score decreased, but the difference was not significant.

### 3.4. Intragroup Comparison of Pretest and Posttest of the Experimental Group

Table 4 shows the longitudinal comparison of the scores of the experimental group on the pretest and the posttest. It is easy to see that the posttest scores of the experimental group differed from the pretest scores, and the differences in the obsessive-compulsive symptoms, depression, anxiety, and hostility factors were very significant. Overall, the mean and factor scores of the SCL-90 factors decreased in the posttest group, with all factors scoring below 2, indicating that none of the subjects in the experimental group had psychological disorders in any of the ten SCL-90 domains. The SIG value for obsessive-compulsive symptoms was 0.001 (*p* ≤ 0.01), demonstrating that the difference between the pre- and post-measures of obsessive-compulsive symptoms in the experimental group was highly significant. The mean score for the OCD factor also decreased from 16.77 in the pretest to 14.37, and the factor score decreased from 1.68 ± 0.46 (individual subjects had scores of more than 2 on this factor) to 1.44 ± 0.21. The absence of psychological disorders in this factor for all subjects in the experimental group also indicates a very significant increase in OCD symptoms in the posttest. A well-known approach to the treatment of OCD is the “cognitive behavioural therapy,” which consists of thought blocking and exposure response prevention. Thought blocking involves distracting the patient and exerting external control to block obsessive thoughts and is more effective when combined with relaxation exercises. The practice of Tai Chi Chuan is similar to thought blocking: the continuous practice of Tai Chi Chuan diverts the subject's attention and blocks the compulsive thinking, and it is also an effective relaxation exercise. Before practicing Taijiquan, the subject was asked to keep his mind on the Dantian and eliminate distracting thoughts, so his obsessive thoughts were effectively blocked and his compulsive symptoms were significantly improved.

The SIG values of depression and anxiety factors were 0.000 (*p* ≤ 0.01), which proved that the posttest scores of depression and anxiety factors of the experimental group were significantly higher than those of the pretest. Anxiety factor scores on the posttest of the experimental group were very significantly different from those on the pretest. The mean score of the depression factor decreased from 17.37 to 14.57, and the per capita factor score decreased from 1.34 ± 0.36 to 1.12 ± 0.14, which is lower than 2, indicating that none of the subjects in the experimental group had psychological disorders at the time of the posttest, and the level of the posttest was significantly higher than the level of the pretest. The mean score for the anxiety factor decreased from 14.80 to 11.87, and the per capita factor score decreased from 1.34 ± 0.36 to 1.12 ± 0.17, which was significantly lower than 2, indicating that none of the subjects in the experimental group had a psychological disorder at the posttest, and the posttest level was significantly higher than the pretest level. Taijiquan is a traditional fitness boxing method that combines physical exercise, breathing, and mental regulation and can effectively improve the physical and mental health of the practitioners. On this platform, the subjects were able to fully release the accumulated psychological stress by communicating with each other, learning together, laughing together, and working together, thus suppressing bad psychology, promoting psychological health, and improving depression and anxiety. Second, Taijiquan is a low- to medium-intensity aerobic exercise that requires the practitioner to learn to be still and transform the mood in stillness, so the subject can focus on the gongfu and eliminate distractions, which will help improve the subject's anxiety and depression. Apart from the fact that the gongfu and mood of Taijiquan can improve depression and anxiety, the cultural connotation of Taijiquan itself can also effectively promote the mental health of the subjects and improve their depression and anxiety. In addition to mastering the techniques of Taijiquan, the subjects were also asked to learn about the cultural background of Taijiquan and to spend their spare time learning about the historical background of Taijiquan. The profound cultural background of Taijiquan will help the subjects to get in touch with the profound history and culture of China, thus cultivating their traditional culture and enriching their life after school, and to a certain extent, crowding out the bad psychology of the subjects in their life and study. After learning about the cultural background of Taijiquan, the subjects communicated and discussed with each other and promoted it to others, all of which could promote communication between the subjects and others, thus improving the level of depression and anxiety of the subjects.

The SIG value for the hostility factor was 0.001(*p* ≤ 0.01), indicating that the difference between the pre- and posttest hostility factors in the experimental group was highly significant. The mean per capita factor score for the hostility factor decreased from 8.774 to 7.23, and the per capita factor score decreased from 1.46 ± 0.37 to 1.20 ± 0.27. The pretest per capita factor scores showed that all subjects in the experimental group did not have psychological disorders in the area of hostility, while the posttest per capita factor scores was significantly lower than 2, indicating that the posttest level was significantly better than the pretest level. Hostility is mainly due to subjectivity, prejudice, and an excessive psychological defence mechanism, and the practice of Taijiquan is effective in improving this psychological problem.

This will eliminate their prejudices and even their psychological problems of bigotry. Second, the practice of Taijiquan also adds to the subject's ability to interact with others. When practicing Taijiquan, the subjects learn to be calm and peaceful at all times and increase sincere communication between them. It also increases sincere communication between the subjects, allowing them to let go of their differences and defences, thus reducing this excessive psychological defence mechanism. This will reduce this excessive psychological defence mechanism. Therefore, the posttest hostility scores of the experimental group were significantly better than the pretest hostility scores.

The mean total score of the experimental group decreased from 129.73 to 115.73, which means that the mean total score decreased by 14 points. The significance of the sign is 0.001 (*p* ≤ 0.01), which means that the difference in mean scores is highly significant. Total posttest scores were significantly higher than pretest scores, as there were significant differences in SCL-90 posttest scores for obsessive-compulsive symptoms, depression, anxiety, and hostility, with significant increases in each factor. Scores for the other factors also decreased but did not reach the threshold of significance. The increase in total scores also suggests that practicing Tai Chi Chuan improves the overall mental health of participants [19, 20].

After practicing Taijiquan, the participants' obsessive-compulsive symptoms, depression, anxiety, and hostility all showed significant improvements. This suggests that Tai Chi Chuan can reduce students' psychological stress, provide them with appropriate psychological care, eliminate their undesirable psychology in life and study, and effectively improve their psychological health. In addition, the effect of Tai Chi Chuan on depression and the improvement of delusional disorder were stronger in females than in males. The results confirmed the hypothesis that “Taijiquan improved students' mental health and reduced depression and anxiety,” but the hypothesis that “the effects of Taijiquan on anxiety and depression were stronger in males than in females” was not confirmed. There was no significant gender difference in the improvement of anxiety, while the improvement of paranoia was significantly stronger in females than in males.

## 4. Conclusion

Starting from traditional martial arts and taking Taijiquan as an example, this article mainly studies the influence of Taijiquan on the mental health of college students. This article first introduces the objectives and research methods of this article, and then determines the number and specific scope of research through experimental design and operation. Finally, the experimental results and analysis show that Taijiquan, as an item in traditional martial arts, can play a significant role in the mental health of college students. This article only takes Taijiquan in traditional martial arts as an example to study, which has certain limitations. Later, I hope to expand the research scope of traditional martial arts and study more about the psychological health of college students.

## Figures and Tables

**Table 1:** Comparison of pretest SCL-90 data of the experimental control group.

Gene	Group	N	Share out equally	Per capita factor points (M ± SD)	Sig
Somatization	Experimental group	30	14.47	1.21 ± 0.24	0.309
	Control group	30	15.20	1.27 ± 0.22	

Forced symptoms	Experimental group	30	14.37	1.44 ± 0.21	0.079
	Control group	30	15.37	1.54 ± 0.22	

Sensitive to interpersonal relationship	Experimental group	30	13.01	1.46 ± 0.32	0.115
	Control group	30	11.73	1.30 ± 0.41	

Blues	Experimental group	30	14.57	1.12 ± 0.14	0.001^*∗∗*^
	Control group	30	16.23	1.25 ± 0.14	

Inquietude	Experimental group	30	11.87	1.19 ± 0.14	0.000^*∗∗*^
	Control group	30	14.23	1.42 ± 0.12	

Antagonize	Experimental group	30	7.23	1.21 ± 0.25	0.046^*∗*^
	Control group	30	8.13	1.36 ± 0.32	

Consternation	Experimental group	30	8.37	1.20 ± 0.27	0.119
	Control group	30	9.20	1.31 ± 0.31	

Stubborn	Experimental group	30	7.80	1.30 ± 0.22	0.924
	Control group	30	7.77	1.30 ± 0.23	

Psychiatric sex	Experimental group	30	13.93	1.39 ± 0.19	0.945
	Control group	30	13.90	1.39 ± 0.18	

Other	Experimental group	30	10.03	1.43 ± 0.21	0.436
	Control group	30	9.70	1.39 ± 0.25	

TP	Experimental group	30	115.73		0.104
	Control group	30	121.47		

*Note*. ^*∗*^ indicates *p*(Sig) ≤ 0.05, significant difference; ^*∗∗*^ indicates *p*(Sig) ≤ 0.01, highly significant difference.

**Table 2:** Comparison of SCL-90 data in the posttest of the experimental control group.

Gene	Group	N	Share out equally	Per capita factor points (M ± SD)	Sig
Somatization	Experimental group	30	15.73	1.31 ± 0.24	0.718
	Control group	30	15.43	1.29 ± 0.29	

Forced symptoms	Experimental group	30	16.77	1.68 ± 0.46	0.743
	Control group	30	16.37	1.64 ± 0.48	

Sensitive to interpersonal relationship	Experimental group	30	13.13	1.46 ± 0.29	0.722
	Control group	30	12.83	1.43 ± 0.42	

Blues	Experimental group	30	17.37	1.34 ± 0.36	0.909
	Control group	30	17.20	1.32 ± 0.50	

Inquietude	Experimental group	30	14.80	1.48 ± 0.39	0.791
	Control group	30	15.03	1.50 ± 0.29	

Antagonize	Experimental group	30	8.77	1.46 ± 0.37	0.282
	Control group	30	8.17	1.36 ± 0.34	

Consternation	Experimental group	30	9.07	1.30 ± 0.34	0.541
	Control group	30	8.67	1.24 ± 0.33	

Stubborn	Experimental group	30	8.13	1.36 ± 0.34	0.953
	Control group	30	8.17	1.36 ± 0.38	

Psychiatric sex	Experimental group	30	14.80	1.48 ± 0.39	0.677
	Control group	30	14.40	1.44 ± 0.35	

Other	Experimental group	30	11.17	1.60 ± 0.47	0.225
	Control group	30	10.23	1.46 ± 0.36	

TP	Experimental group	30	129.73		0.641
	Control group	30	126.50		

*Note*. ^*∗*^ indicates *p*(Sig) ≤ 0.05, significant difference; ^*∗∗*^ indicates *p*(Sig) ≤ 0.01, highly significant difference.

**Table 3:** Comparison of SCL-90 data in the control group pre- and posttests.

Gene	Group	N	Share out equally	Per capita factor points (M ± SD)	Sig
Somatization	Experimental group	30	15.43	1.29 ± 0.29	0.467
	Control group	30	15.20	1.27 ± 0.22	

Forced symptoms	Experimental group	30	16.37	1.64 ± 0.48	0.177
	Control group	30	15.37	1.54 ± 0.22	

Sensitive to interpersonal relationship	Experimental group	30	12.83	1.43 ± 0.42	0.055
	Control group	30	11.73	1.30 ± 0.41	

Blues	Experimental group	30	17.20	1.32 ± 0.50	0.389
	Control group	30	16.23	1.25 ± 0.14	

Inquietude	Experimental group	30	15.03	1.50 ± 0.29	0.156
	Control group	30	14.23	1.42 ± 0.12	

Antagonize	Experimental group	30	8.17	1.36 ± 0.34	0.925
	Control group	30	8.13	1.36 ± 0.32	

Consternation	Experimental group	30	8.67	1.24 ± 0.33	0.247
	Control group	30	9.20	1.31 ± 0.31	

Stubborn	Experimental group	30	8.17	1.36 ± 0.38	0.312
	Control group	30	7.77	1.30 ± 0.23	

Psychiatric sex	Experimental group	30	14.40	1.44 ± 0.35	0.264
	Control group	30	13.90	1.39 ± 0.18	

Other	Experimental group	30	10.23	1.46 ± 0.36	0.228
	Control group	30	9.70	1.39 ± 0.25	

TP	Experimental group	30	126.50		0.102
	Control group	30	121.47		

*Note*. ^*∗*^ indicates *p*(Sig) ≤ 0.05, significant difference; ^*∗∗*^ indicates *p*(Sig) ≤ 0.01, highly significant difference.

**Table 4:** Comparison of SCL-90 data in the pretest and posttest of the experimental group.

Gene	Group	N	Share out equally	Per capita factor points (M ± SD)	Sig
Somatization	Experimental group	30	15.73	1.31 ± 0.24	0.078
	Control group	30	14.77	1.21 ± 0.24	

Forced symptoms	Experimental group	30	16.77	1.68 ± 0.46	0.001^*∗∗*^
	Control group	30	14.37	1.44 ± 0.21	

Sensitive to interpersonal relationship	Experimental group	30	13.13	1.46 ± 0.29	0.949
	Control group	30	13.10	1.46 ± 0.32	

Blues	Experimental group	30	17.37	1.34 ± 0.36	0.000^*∗∗*^
	Control group	30	14.57	1.12 ± 0.14	

Inquietude	Experimental group	30	14.80	1.34 ± 0.36	0.000^*∗∗*^
	Control group	30	11.87	1.12 ± 0.14	

Antagonize	Experimental group	30	8.77	1.46 ± 0.37	0.000^*∗∗*^
	Control group	30	7.23	1.21 ± 0.25	

Consternation	Experimental group	30	9.07	1.30 ± 0.34	0.127
	Control group	30	8.37	1.20 ± 0.27	

Stubborn	Experimental group	30	8.13	1.36 ± 0.34	0.288
	Control group	30	7.80	1.30 ± 0.22	

Psychiatric sex	Experimental group	30	14.80	1.48 ± 0.39	0.238
	Control group	30	13.93	1.39 ± 0.19	

Other	Experimental group	30	11.17	1.60 ± 0.47	0.065
	Control group	30	10.03	1.43 ± 0.21	

TP	Experimental group	30	129.73		0.001^*∗∗*^
	Control group	30	115.73		

*Note*. ^*∗*^ denotes *p*(Sig) ≤ 0.05, significant difference; ^*∗∗*^ denotes *p*(Sig) ≤ 0.01, highly significant difference.

## Data Availability

The data that support the findings of this study are available from the corresponding author upon request.
